# Mental Health Identification of Children and Young Adults in a Pandemic Using Machine Learning Classifiers

**DOI:** 10.3389/fpsyg.2022.947856

**Published:** 2022-07-29

**Authors:** Xuan Luo, Youlian Huang

**Affiliations:** School of Pre-school Education, Yichun Early Childhood Teachers College, Yichun, China

**Keywords:** machine learning, COVID-19, artificial intelligence, mental health, feature selection, mood state, clustering

## Abstract

COVID-19 has altered our lifestyle, communication, employment, and also our emotions. The pandemic and its devastating implications have had a significant impact on higher education, as well as other sectors. Numerous researchers have utilized typical statistical methods to determine the effect of COVID-19 on the psychological wellbeing of young people. Moreover, the primary aspects that have changed in the psychological condition of children and young adults during COVID lockdown is analyzed. These changes are analyzed using machine learning and AI techniques which should be established for the alterations. This research work mainly concentrates on children's and young people's mental health in the first lockdown. There are six processes involved in this work. Initially, it collects the data using questionnaires, and then, the collected data are pre-processed by data cleaning, categorical encoding, and data normalization method. Next, the clustering process is used for grouping the data based on their mood state, and then, the feature selection process is done by chi-square, L1-Norm, and ReliefF. Then, the machine learning classifiers are used for predicting the mood state, and automatic calibration is used for selecting the best model. Finally, it predicts the mood state of the children and young adults. The findings revealed that for a better understanding of the effects of the COVID-19 pandemic on children's and youths' mental states, a combination of heterogeneous data from practically all feature groups is required.

## Introduction

The World Health Organization (WHO) confirmed the new coronavirus (COVID-19) as its source of pneumonia in Wuhan, China, in December 2019, and proclaimed COVID-19 a pandemic on 11 March 2020 (Ntakolia et al., 2022). About 184 nations enacted strict precautions to control the growth of COVID-19 between 31 December 2019 and 4 May 2020, including lockdown limitations and quarantined periods, resulting in economical, ecological, and mental health problems. The lockdown tactics helped governments to reduce the spread of COVID-19, but the rise of mental health problems is highly concerning. Furthermore, the lockdown is still in effect, and the total academic sector has been affected, with schools, colleges, and institutions facing partial or complete closures, so both academic and non-academic activities are severely impacted (Demir et al., 2022). However, the lockdown is enforced and maintained to prevent the virus from spreading, and a slew of negative consequences have emerged. To begin with, all academic and non-academic events have been suspended. Pupils are becoming bored due to the closure of academic institutions, and the drive for gaining information to be successful in a positive manner is dwindling.

The effect of COVID-19 as well as its limitation rules on the researched group has been investigated in a number of studies (McKune et al., 2021; Qin et al., 2021; Błaszczyk et al., 2022). Multivariable logistic regression models were used in many research to: (i) examine the possible risk factors defined as self-emotional problems (Ren H. et al., 2021) and (ii) compare the impact of COVID-19 assessments (Gomathi et al., 2021).

Even during a disease outbreak, binomial or binary logistic multiple regressions have been used to: (i) recognize difficulty sleeping between many adolescents and young adults (12–29 years) (Islam et al., 2020; Zhou et al., 2020), (ii) evaluate anxiety and depression between many college students (Gomathi et al., 2020; Yeasmin et al., 2020), and (iii) investigate the risk of developing depression between many children as well as the potential connection to COVID-19 (Garcia de Avila et al., 2020). Univariate logistic regression analysis was employed in other research focused on youth to detect psychological disorders (Shanmugam et al., 2017; Liang et al., 2020). Then, during the COVID-19 epidemic among University students, hierarchical logistic regression models were employed to investigate characteristics linked to mental health concerns (Ma et al., 2020). The relationship among COVID-19 anxiety and problems in children and teenagers was investigated using modified logistic regression analysis (Ma et al., 2020).

The results of previous studies introduced above centered on Chinese regions and University students and also used conventional regression algorithms to detect correlation coefficients between risk variables and mental health issues, such as logistic regression and chi-square examinations (Ge et al., 2020; Rens E. et al., 2021; Sciberras et al., 2022), although only very few were using machine learning techniques. Moreover, no study focusing on children and teens with identified mental problems has been conducted to their understanding. As a result, this research proposed the establishment of such an understandable machine learning pathway to understand the implications and effects of Greece's first lockdown on the mental health of children and teenagers.

The main contribution of the proposed work is given below:

- In this work, a *post hoc* explainability model is used for detection and it identifies the mental health of youths and adults during the lockdown in Greece,
- Susceptible, Infected, Recovered, and Deceased (SIRD) automatic calibration model effectively detects the mood states and reduces the computation cost.
- For the feature selection process, it uses chi-square, L1-Norm, and ReliefF method, which efficiently selects the features for detecting mental health.

The rest of our research article is written as follows: Section Related Work discusses the related work on various COVID-19 lockdown scenarios and mental health. Section Proposed Method shows the algorithm process and general working methodology of the proposed work. Section Result Analysis evaluates the implementation and results of the proposed method. Section Conclusion concludes the work and discusses the result evaluation.

## Related Work

Primarily, during the COVID-19 pandemic, a multivariable logistic regression method was used to test connections between socio-demographic characteristics and mental health issues in Chinese teenagers. There were 8,079 Chinese students aged 12 to 18 in the community. The Patient Health Questionnaire (PHQ-9) and the Generalized Anxiety Disorder (GAD-7) questionnaire were used to obtain information to assess symptoms of depression and anxiety. Female students as well as those with top grades were shown to have a higher probability of reporting mental health symptoms (Chakraborty and Maity, 2020).

Similarly, throughout COVID-19, secondary research was completed on the psychological health of Chinese children between the ages of 7–15 years, with a number of 668 families from various provinces of China. The statistical analyses were performed using multiple logistic regression assessment to determine the elements that make a contribution to Chinese children's support and mental health, and it was discovered that public schools and the provincial capital of beginnings were the important considerations associated with treating PTSD, with the majority of individuals showing a better viewpoint regarding online learning (WHO, 2020). The author used information from the General Health Questionnaire (GHQ-12), the PTSD Checklist—Civilian Version (PCL-C), or the Adverse Behavioral Strategies Scale to investigate the impact of COVID-19 on juvenile mental illness in China.

The effectiveness of simulation using epidemiological models (SIR, SEIRV, etc.) was also examined, as was the discovery of design variables (Bonardi et al., 2020; Vindegaard and Benros, 2020; Abas et al., 2021; Ma et al., 2021), which are critical for successful modeling fits into actual data. Furthermore, the contemporary estimating methodology allows the study of design variables as they emerge and continuous updating of their estimates, thanks to the tremendous development in processing capacity in recent years. For instance, (Vizheh et al., 2020) examined several time-series approaches to forecast the number of actual COVID-19 incidences and mortality in Chile. In (Penner et al., 2021) employed a Bayesian method again for an agent-based system. Finally, Prati and Mancini (2021) examined deep learning approaches (based on LSTM neural networks).

The relationship between socio-demographic characteristics and COVID-19-related characteristics, as well as their impact on sadness, tension, and pressure among teenagers in Spain, was investigated (Masten, 2021). A final tally of 523 adolescents (13–17 years old) finished the Depressive episodes, Nervousness, and Anxiety Scale (DASS-21) and the Oviedo Infrequency Scale (INFO-OV), with findings denoting those girls who worked knowingly and willingly and decided to stay home more commonly, and were much more inclined to display the signs of depression, anxiousness, and strain. Furthermore, when performing COVID-19 study, the researchers discovered a link between mental anguish and chronic stress. Finally, those in a romantic connection, as well as those who had previously been afflicted with COVID-19, were much more likely to also have better psychological health. A summary of research on the first COVID-19 pandemic is stated in Table 1.

**Table 1:** A summary of research on the first COVID-19 pandemic, which included teens and young people.

**Author**	**Region**	**Number of Populations**	**Focus**	**Methodologies used**
Ren Z. et al. (2021)	China	After the reopening of the institution, 478 college students	COVID-19's psychological influence was investigated.	Multivariate logistic regression
Cost et al. (2021)	Canada	One thousand thirteen infants and young people between the ages of 6 and 18, even without prior illnesses	To assess the impact of COVID-19 on mental wellbeing.	Multinomial logistic regression
Garcia de Avila et al. (2020)	Brazil	6–12 years old: 157 females and 132 boys	To see how common anxiousness was there during COVID-19.	Logistic regression
Yeasmin et al. (2020)	Bangladesh	Three hundred eighty-four families with at minimum one child under the age of eight	Detecting psychological problems during COVID-19	Binary logistic regression
Wathelet et al. (2020)	France	69,054 college students in France	COVID-19-related mental health disorders will be investigated.	Multivariate logistic regression
Sciberras et al. (2022)	Australia	Families of 213 ADHD-diagnosed children and adolescents ages 5 to 17 years old	To determine the COVID-19 limitations' effect	Adjusted logistic regression analyses

The network reliability is discussed by Ansari and Malekshah (2019). Security of the system is the key assessment (Malekshah and Javad, 2021) which is implemented for environmental-related data distribution. Deep reinforcement learning (Malekshah et al., 2022) is used for distributing the power in the dynamic network with high reliability.

The limitations of the existing work are studied above. The main issue is that some techniques fail to estimate real situations before taking statistics. The situation in the sense is that if some people are infected with COVID, then the families have high mental pressure. It is a different scenario. Also, the accuracy of the prediction is not as expected.

## Proposed Method

In this work, we concentrated on the marginalized populations of children and teenagers to forecast the effect of COVID-19 and the first lockdown implemented in Greece from 23 March to 4 May 2020. The Hellenic COVID-19 impact survey (HOPE) information is used, in a large study of parents with children who were planning to attend CAMHS in Greece each year even before the global epidemic (1 March 2019 to 1 March 2020). The proposed work consists of six stages. Initially, the data are collected through a questionnaire. Then, the collected information is pre-processed. Then, the clustering process is done, and feature selection is based on chi-square, L1-Norm, and ReliefF. Next, it uses the automatic calibration method Susceptible, Infected, Recovered, and Deceased (SIRD) along with the machine learning models that were used for evaluation. Finally, a *post-hoc* explainability helps to detect the best feature using the SHAP model. Figure 1 shows the overall architecture of the proposed model.

**Figure 1:** Architecture of proposed method.

### Collection of Data

Children who used CAMHS services were recruited to effectively gather data and create the dataset. This research included 744 children who had their parents (738 parents) complete an online survey on their own. Through 8 May and 1 June 2020, this process was performed. The questionnaire asked about demographic data as well as the parent's assessment of their patient's care 3 months (3 m) well before lockdown and 2 weeks (2 w) following the very first lockdown in Greece.

### Pre-processing

There was no requirement for data imputation because the final dataset had no missing values for categorical or numerical variables. Moreover, the dataset was standardized, which is a frequent prerequisite for many ML classifiers.

#### Data Cleaning

Removing the dataset is the first step in processing it, and it entails carefully removing redundant items and attributes. To start, several categorical variables in the dataset must be deleted for the concerns of confidentiality.

#### Categorical Encoding

Age, parent, symptoms, and all data points in the dataset must be encoded. Encoding is essential if ML techniques demand numerical data and therefore can handle categorical variables. This study employed one-hot encoding, which creates “dummy” values for each non-numeric attribute's potential classes.

#### Data Normalization

Most of the items in the data are integers, as noted previously. A handful of these features were also obtained with the help of additional measuring instruments. The performance of the algorithms may be harmed if these attributes are handled without normalization. Normalization is needed to dynamically expand all numerical values into a range between 0 and 1.

(1) $$\begin{array}{r} NOR=\frac{Val-MIN}{MAX\;} \end{array}$$

Here, MAX and MIN are the maximum and minimum column values, respectively. Equation 2 shows the normalization formula.

### Clustering Process

Several clustering methods were compared. Mini Batch K-Means (Peng et al., 2018), spectral clustering (Von Luxburg, 2007), ward (Ward, 1963; Murtagh and Legendre, 2014), average linkage (Yim and Ramdeen, 2015), balanced iterative reducing and clustering utilizing hierarchies (Birch) (Anchang et al., 2016), and Jenks natural breaks optimization approach (Jenks) (North, 2009; Zhang et al., 2021) were used in the clustering process. The occurrences of the parameter mood change, which reflects the changes in mood state, were clustered.

The parameters such as worry, sorrow, anxiety, uneasiness, anhedonia, isolation, irritation, focus, weariness, and rumination are used to construct the emotional condition rating before and during the lockdown. The difference in mood state throughout the last 2 weeks and 3 months until the first lockdown in Greece is the variation in emotional experience. As a result, a negative value for the forecasted variable mood change suggests that the user's mood state score has improved overall, whereas a positive value suggests that the user's attitude condition score has worsened on the whole. Results near to 0 indicate that the subject's mood state score did not change during the lockdown. Figure 2 shows the clustering methods used.

**Figure 2:** Clustering methods used.

### Feature Selection

The ReliefF, chi-square, and L1-Norm algorithms were used in the feature selection procedure because of their usefulness in diagnosing diseases and categorization difficulties. ReliefF is an approximation of the traditional relief that, thanks to its noise resistance increase, can cope with multiclass difficulties and is thus regarded as ideal again for the present healthcare multiclassification challenge. Figure 3 shows the feature selection methods used.

**Figure 3:** Feature selection method used.

#### Chi-Square

A significant feature sfi is picked in the chi-square methods based on its association with a Chj class, and the differentiating capability of features sfi followed Chj class is determined using the formula:

(2) $$\begin{array}{r} X^{2}\left(sf_{i},Ch_{j}\right)=\frac{M\times {\left(a_{ij}d_{ij}-b_{ij}c_{ij}\right)}^{2}}{\left(a_{ij}+b_{ij}\right)\times \left(a_{ij}+c_{ij}\right)\times \left(b_{ij}+c_{ij}\right)\times \left(c_{ij}+d_{ij}\right)} \end{array}$$

where M represents the number of observations in the Chj class that contain feature sfi is aij, and the number of samples in the Chj class that do not have feature sfi is bij (Anchang et al., 2016). The sample in the Chj class that includes features sfi is aij, whereas the number of samples in the Chj class that do not have feature sfi is bij (Guru et al., 2018). The number of observations with characteristic sfi which are not in the Chj class is given by cij. Finally, dij is the sample size that does not have either as the feature ti or even the Chj class.

#### Relief Algorithm

When targeted categories are multiclass categorical variables, the ReliefF method calculates the predictive weight. Predictors who show various ratings to neighbors in the same class are punished, but predictors who give the same scores to neighbors in the very same class are encouraged (Tuncer et al., 2020). The predictor variables (WEj) in the ReliefF method are originally set to 0. The ReliefF algorithm selects a randomized forecast (xs) on a regular basis, then determines the k-nearest forecasts to xs within every class, and modifies every nearest neighbor (xt) (Demir et al., 2020; Turkoglu, 2021). If somehow the xs and xt classes would be the same, all of the forecasters' values (Pi) are as continues to follow:

(3) $$\begin{array}{r} WE_{i}^{j}=WE_{i}^{j-1}-\frac{\Delta_{j}\left(x_{s},x_{t}\right)}{n}d_{st} \end{array}$$

If such x_s_ and x_t_ categories vary, all of the predictors' values (P_i_) were just as described as follows:

(4) $$\begin{array}{r} WE_{i}^{j}=WE_{i}^{j-1}=\frac{Py_{s}}{1-Py_{t}}.\frac{\Delta_{j}\left(x_{s},x_{t}\right)}{n}d_{st} \end{array}$$

where py_s_ denotes the prior possible of a category toward which x_s_ corresponds, py_t_ indicates the prior probability of the category toward which x_q_ originally belonged, n represents the total of repetitions modified by updating, and Δi(x_s_, x_t_) is the differential with in scores of a predictors Pj among occurrences x_s_ and x_t_. The P_i_, Δi(x_s_, x_t_), could be described as follows for preciseness:

(5) $$\begin{array}{r} i\left(x_{s},x_{t}\right)=\{\begin{array}{c} 0,\;x_{s\left(i\right)}=x_{q\left(i\right)}\\ 1\;x_{s\left(i\right)\neq x_{q\left(i\right)}} \end{array} \end{array}$$

(6) $$\begin{array}{r} dis_{st}=\frac{dis_{st}^{\sim }}{\sum_{t=1}^{l}dis_{st}^{\sim }} \end{array}$$

(7) $$\begin{array}{r} dis_{st}^{\sim }=e^{-{\left(rank\left(s,t\right)/sigma\right)}^{2}} \end{array}$$

Here, rank(s,t) would be the position of the t^th^ information among the s^th^ observation's closest neighbors, arranged by proximity. The value l represents the nearest neighbors.

#### L1-Norm SVM

The cost variable for both the features range of choice L1-Norm SVM (Haq et al., 2019) was used to compute the amount of variables. The continuity formula represents the dataset using m elements:

(8) $$\begin{array}{r} SE=::\left(x_{i},y_{i}\right)|x_{i}\in Rf^{n},y_{i}\in ::-1,1;;{;;}_{i=1}^{k} \end{array}$$

If x_i_ would be the i^th^ samples with n characteristics and a class label, y_i_ is the ${\text{y}}_{\text{i}}^{\text{th}}$ sample (y_i_).

Together in the two-class classification task (Equation 10), the SVM finds the separation of the hyperplane which maximizes the boundary length.

(9) $$\begin{array}{r} y_{i}=\left(Wx_{i}-b\right)\geq 1,i=1,\ldots ..,k \end{array}$$

(10) $$\begin{array}{r} min\frac{1}{2}||W{\left|\right|}^{2} \end{array}$$

As just an outcome of sparse answers, Bradley and Mangasarian utilized Equation (10) by recognizing Equation (11) as a restriction for feature selection-based L1-Norm SVM.

(11) $$\begin{array}{r} \min||W||+B\sum_{i-1}^{k}\max{\left(0.1-y_{i}\left(\alpha^{T}x_{i}+b\right)\right)}^{2} \end{array}$$

here, α the weight matrix produced by the optimizing multipliers seems to be the Lagrange (Guo et al., 2017).

Furthermore, the size of the feature set is measured by the amount of the C variable in Equation (11).

### Data Classification

For data classification, there are seven popular classifiers used and evaluated to overcome the specified multiclass classification issue: random forest (RF), multilayer perceptron (MLP), eXtreme Gradient Boosting (XG Boost), logistic regression (LR), support vector machine (SVM), k-nearest neighbor (KNN), and decision trees (DTs). The accepted methods are often utilized for clinical classification tasks, and they include tree-based, linear, and neural network prediction models.

#### Random Forest

A decision tree forecasts future occurrences using several classifiers instead of a single classifier to arrive at a precise and reliable forecast. RF creates an enormous amount of decision trees. Every decision tree produces a class forecast, and the model's prediction seems to be the category with more scores.

#### Extreme Gradient Boosting (XG Boost)

The eXtreme Gradient Boosting is a versatile and trimming gradient-boosting software program. Gradient boosting is a technique that uses a fresh method to forecast the residuals of past versions which are then combined to form the prediction accuracy. While introducing additional models, it utilizes a gradient descent approach to minimize loss.

#### Multilayer Perceptron

Multilayer perceptron is the most frequent neural network in the area of artificial neural networks (ANNs). MLP uses a supervised learning technique to create a non-linear prediction system. It has several layers, including an input layer, an output layer, and the hidden layers. As a result, MLP is a multilayer feedforward neural network in which data are transported unidirectionally from source to the destination layer *via* the hidden layers.

#### Logistic Regression

The link between data and binary dependent variables is described by a mathematical model. The logistic function f (x) = 1/1+e-x is used in the model, with x (-∞, ∞+) and 0 ≤ f (x) ≤ 1. As a result, compared to the value of x, the framework is meant to explain the data in an A-shaped graph with a probability between 0 and 1.

#### SVM

Support vector machine is a supervised learning model that uses the VC theory statistical learning approach. SVM aims to build a binary classifier, the hyperplane, among two categories that allow for label prediction through one or even more extracted features while maximizing the separation between the nearest distance of every class, termed weight vector, and the hyper-plane.

#### KNN

K-nearest neighbor is a non-parametric classification approach that attempts to categorize an unknown substance based on its neighbors' known categorization.

#### Decision Trees

DTs are sequencing designs that integrate a series of simple tests systematically. Every test was used to compare a numerical characteristic to a threshold level or a nominal property to a range of outcomes.

### Calibration Using SIRD Model

We looked at two fundamental fractional transmissions of infection theories that can be applied to information combining locally and nationally epidemiological data. The driving concern was whether certain simple models might assist in predicting future trends in daily epidemiology data. The most basic mathematical method to simulate the evolution of communicable diseases is the SIR paradigm (Błaszczyk et al., 2022), which assumes a community of size N split into S vulnerable, I infected, and R removing people. These three parameters are time-dependent and reflect the number of patients in each group at a specific moment in time.

The pattern suggests that mortality is limited to a subgroup of resistance people, as determined by R development, and also that sickness does not quite introduce additional vulnerable persons after recovering. The SIR system is defined by the following set of equations when studied on the time period [a, b] [0, T] even without vital movements (births and deaths).

(12) $$\begin{array}{r} SH^{{}^{\prime }}=-\frac{\beta }{N}SI,\;IN^{{}^{\prime }}=\frac{\beta }{SI}-\gamma I,\;RE^{{}^{\prime }}=\gamma I,\;DE^{{}^{\prime }}=\mu I \end{array}$$

where t ϵ [a, b] seems to be the transmitting frequency (gets to control overall amount of spreading), γ is indeed the recovering sample mean, and R0 = $-\frac{\beta }{\gamma }$ is the fundamental reproductive ratio. Several nations track not just the amount of newly confirmed samples and infected people changing constantly, as well as the number of deaths caused by COVID-19.

The tracking is based on the primary goals of nations where Covid case values are determined by standard systems of government. We introduced three low-level cost features presuming that the series ::y_i_;;${}_{\text{i}}^{\text{n}}=$1 includes numbers corresponding to the case of the original Y ϵ::I, R, D;;, for every sequential day from 1 to n, and that$::{\hat{y}}_{i}{;;}_{i=1}^{n}$ refers to the relating obtained values from the Euler scheme [applicable to (1)] with initial state $\hat{y}$_1_ − *y*_1_.

(13) $$\begin{array}{r} MXSE\left(Y\right)=max_{i=1,\ldots ,n}^{e_{i}^{2}} \end{array}$$

(14) $$\begin{array}{r} MSE\left(Y\right)=\frac{1}{n}\sum_{i-1}^{n}e_{i}^{2} \end{array}$$

(15) $$\begin{array}{r} MAE\left(Y\right)=\frac{1}{n}\sum_{i=1}^{n}|e_{i}| \end{array}$$

(16) $$\begin{array}{r} MAPE\left(Y\right)=\frac{100\%}{n}\sum_{i=1}^{n}|\frac{e_{i}}{y_{i}}| \end{array}$$

The second method assumes that now, the major goal function is influenced by all 3 sections, particularly I, R, and D. It is worth noting that its second option is significantly more computationally demanding. Because each compartment of the system may well have data across distinct categories, the relative error of the proposed low-level cost equations with the exception of the MAPE example may be significantly different. As a result, we were making it easy correct normalization to treat each section identically. Then, have a look at the latest set of services.

(17) $$\begin{array}{r} f_{Y}\left(y\right)=\frac{y-\min_{i=1,\ldots .,n}^{y_{i}}}{\max_{i=1,\ldots ,n}^{y_{i}}-\min_{i=1,\ldots ,n}^{y_{i}}} \end{array}$$

where::y_i_;;${}_{\text{i}}^{\text{n}}=$1 signifies a series of observed Y values from consecutive weeks::1,…, n;;. For divisions I, R, and D, the proposed methods were utilized to rescale not just given numbers but also values acquired from the Euler scheme.

We require a independent benchmarking data variable. Finally fitness correction is evaluated and performance is compared with other optimal solutions of optimization methods. Consequently, one of them might be our first choice. In these trials, we opted to use an R^2^ value to assess the matching quality of low-level cost models that were not described.

(18) $$\begin{array}{r} R^{2}\left(YE\right)=1-\frac{\sum_{i=1}^{n}e_{i}^{2}}{\sum_{i=1}^{n}{\left(y_{i}-y\right)}^{2}} \end{array}$$

This was generally determined using only the Y = D variable. Although we employ many optimization methods, the finest potential segment D forecast is our end objective and that is the primary reason for concentrating on this section of the design.

### *Post-hoc* Explainability

The Shapley Additive exPlanations (SHAPs) are used in this research to evaluate the dataset's characteristics in terms of its effects just on the last machine learning results. SHAP uses a coalitional game model to compute optimal Shapley ratios. These numbers indicate how evenly the impact on the model's predictions is divided across the dataset's characteristics. Next, in terms of explaining how well this forecast was made, SHAP creates a mini-explainer architecture that correlates with just a single-row forecast pairing.

## Result Analysis

Employing healthcare data collected from the dataset, the research framework was used to predict the changes in the emotional experience of children and teens who have been diagnosed with chronic disorders. During a calibration procedure, the best-performing clustering approach is reviewed, and multiple prediction methods are assessed based on the outcomes of the feature selection technique to identify the best-performing depending on the accuracy metric. A *post hoc* explainability study is conducted just on best-performing calibration to obtain a greater understanding and interpretations of the most significant contributing aspects to the model's outputs.

### Environmental Setup

The Silhouette coefficient, the Calinski–Harabasz Index, and the Davies–Bouldin Index are the three clustering determining factors that are integrated. To calculate a cumulative average rating, the normalized values of the assessment criteria are added together. The clustering algorithms were used with standard system parameters from the sklearn.cluster modules (https://scikit-learn.org/stable/modules/classes.html#module-sklearn.cluster, viewed on 1 August 2021), whereas the model variables were seen in Table 2. The feature selection is then conducted just on 3 clusters obtained by the predominant clustering algorithm using ReliefF, L1-Norm, and chi-square.

**Table 2:** Clustering technique's parameter settings.

**Methods**	**Parameter settings**
Spectral clustering	Three classes, arpack eigen solver, and affinities for nearest neighbors
Average linkage	Average linkage, cityblock affinity, and symmetric connection are three kinds.
Mini Batch K-means	Three classes
Ward's hierarchical agglomerative clustering	Symmetric connection, three classes, ward linkage
Birch	Three classes
Jenks	There are three classes, including the lowest value.

The minority classes were classified using a repeating stratification 5-fold cross-validation using grid search using the SMOTE technique—oversampling to the training sample. Components of characteristics with growing complexity were used to assess the predictive model. The reliability of the prediction methods was selected as the method of evaluating their effectiveness.

### Feature Selection

Figure 4 shows the spider graph with the number of attributes from every category for the first 40 characteristics where the greatest result was attained, resulting from ReliefF, chi-square, and L1-Norm. The features are listed in Table 2 (Ntakolia et al., 2022).

**Figure 4:** For the first 40 features in which the greatest result was attained, a spider plot showing the amount of characteristics that correspond to every characteristic group was created.

### Classification and Calibration

The efficiency of the comparison prediction methods for the range of features is shown in Figure 5. Table 3 illustrates the optimum value accuracy of every estimation method employed in the various experiments, as well as the number of characteristics where it was attained.

**Figure 5:** Maximum accuracy for classification methods.

**Table 3:** Maximum accuracy for classification methods.

**Models**	**Maximum accuracy (%)**	**Number of features for maximum accuracy**
Random forest	68.6	44
MLP	59.38	58
XG Boost	72.43	40
Logistic regression	56.74	50
SVM	66.95	49
KNN	53.28	3
Decision trees	52.23	5

We calibrate the XG Boost model using the SIRD model and compare it to current models such as isotonic regression to improve its efficiency. To evaluate the models, we are using the logistic regression loss (Log-loss) as well as the correctness. Table 4 demonstrates the results of using SIRD, and isotonic regression to calibrate the XG Boost classifier.

**Table 4:** Results of using SIRD, isotonic regression to calibrate the XG Boost classifier.

**Models used**	**Log-loss**	**Accuracy**
XG Boost	1.196	68.98
XG Boost+Isotonic	0.513	73.12
XG Boost+SIRD	0.352	78.98

Figure 6 measures the variation in projected probability on sample material following isotonic regression and SIRD calibration, correspondingly. True categories 0, 1, and 2 are represented by the red, green, and blue hues of an arrow, accordingly. Class 0, class 1, and class 2 participants, alternately, have a negative, neutral, or positive alteration in their emotional experience. The calibration charts for every class above all others are shown in Figures 7–9.

**Figure 6:** Following calibration using isotonic and SIRD model, change in expected probability on test samples.

**Figure 7:** XG Boost classifier calibration graph for class 0.

**Figure 8:** XG Boost classifier calibration graph for class 1.

**Figure 9:** XG Boost classifier calibration graph for class 3.

## Discussion

### Feature Selection

The findings indicated that social life factors had a considerable impact on predicting outcomes (Table 1, Figure 4). Furthermore, the spider graph (Figure 4) shows that nine characteristics from people's social groups were in the top 40 most important qualities. Moreover, with six elements inside the attribute selection subgroup, everyday routines are the second least important category. Finally, behavioral and demographic effects each provide five characteristics. Health treatment, sleep pattern, medical problems, home life, and private life are the other characteristics (Figure 4). The foregoing findings clearly show that characteristics in all areas are required to properly predict the effect of COVID-19 on the emotional responses of children and teenagers.

### *Post-hoc* Explainability

The mood change, or the changing in emotional experience prior to actually and after the first lockdown in Greece, was chosen as the predicted variable in this research. The findings revealed that the family's perspectives as to whether the COVID-19 emergency caused changes for the better in their child's growth (2 w positive), their family life (2 w relationships family), and their psychological health assessment prior to the COVID-19 emergency (3 m tv) were all strongly linked to a child's emotional experience. Furthermore, during the 3 months prior to and 2 weeks just after lockdown, the amount of time spent watching television or using electronic devices by children increased significantly. As a result, we can see that lockdown had a harmful effect on children who did not originally spend significant time watching television but now do. It is worth noting that the first diagnostic given by a healthcare practitioner played a significant effect in the child's personality change.

## Conclusion

An understandable machine learning pathway was developed in this work to study and identify its most essential factors related to the emotional state shifts of children and teens throughout Greece's first lockdown. The focus of this research is to discover and explain the elements that influenced the psychological health of the studied group throughout the first COVID-19-related lockdown using the chosen ML workflow. As a result, the issue was defined as a three-class classification issue to detect the variations in the emotional experience of the persons under investigation. Persons with positive (class 0) and negative (class 2) mood alterations, as well as those with no major change in emotional experience, were divided into classes (class 1). To find the optimum clustering approach and prediction model for this topic, a detailed comparative evaluation was conducted. The Jenks approach was chosen for clustering, followed by feature selection using ReliefF, chi-square, and L1-Norm. After that, the best-performing prediction, the XG Boost with SIRD and isotonic model, was utilized for calibration and a *post-hoc* explainability study to validate the key characteristics that contributed to a model's estimate places. Furthermore, the impact of every characteristic on the various classes was discussed.

We can conclude that the positive developments in a child's life as a result of the first lockdown—family relationships, time was spent watching TV, parenting practices assessment of the child's mental health, and stress created by COVID-19 restrictions—could play a critical role in the change in the child's mood state. These findings are consistent with those of previous research that used pre-pandemic healthcare instances or population-based groups of children who are at risk of transitioning between subclinical to medically severe levels of psychosis. The findings of this study can be effectively employed for the primary requirements of physicians which can be properly prepared for future emergencies or restrictions.

## Data Availability Statement

The original contributions presented in the study are included in the article/supplementary material, further inquiries can be directed to the corresponding author/s.

## Author Contributions

Both authors listed have made a substantial, direct, and intellectual contribution to the work and approved it for publication.

## Funding

This work was supported by the Social Science Research Planning Project of Jiangxi Province, China, “The Influence of Moral Emotion on Online Helping Behavior of College Students” (19JY46).

## Conflict of Interest

The authors declare that the research was conducted in the absence of any commercial or financial relationships that could be construed as a potential conflict of interest.

## Publisher's Note

All claims expressed in this article are solely those of the authors and do not necessarily represent those of their affiliated organizations, or those of the publisher, the editors and the reviewers. Any product that may be evaluated in this article, or claim that may be made by its manufacturer, is not guaranteed or endorsed by the publisher.
